The article "Liposomes: Structure, Biomedical Applications, and Stability Parameters With Emphasis on Cholesterol" was retracted in 2023. Reasons: signs of a paper mill; concerns about the authorship.

# Liposomes: Structure, Biomedical Applications, and Stability Parameters With Emphasis on Cholesterol

**DOI:** 10.3389/fbioe.2021.705886

**Published:** 2021-09-09

**Authors:** Pooria Nakhaei, Ria Margiana, Dmitry O. Bokov, Walid Kamal Abdelbasset, Mohammad Amin Jadidi Kouhbanani, Rajender S. Varma, Faroogh Marofi, Mostafa Jarahian, Nasrin Beheshtkhoo

**Affiliations:** ^1^ School of Medicine, Tehran University of Medical Sciences, Tehran, Iran; ^2^ Department of Anatomy, Faculty of Medicine, Universitas Indonesia, Depok, Indonesia; ^3^ Cipto Mangunkusumo Hospital, The National Referral Hospital, Central Jakarta, Indonesia; ^4^ Master’s Programme Biomedical Sciences, Faculty of Medicine, Universitas Indonesia, Depok, Indonesia; ^5^ Institute of Pharmacy, Sechenov First Moscow State Medical University, Moscow, Russia; ^6^ Laboratory of Food Chemistry, Federal Research Center of Nutrition, Biotechnology, and Food Safety, Moscow, Russia; ^7^ Department of Health and Rehabilitation Sciences, College of Applied Medical Sciences, Prince Sattam Bin Abdulaziz University, Al Kharj, Saudi Arabia; ^8^ Department of Physical Therapy, Kasr Al-Aini Hospital, Cairo University, Giza, Egypt; ^9^ Department of Medical Nanotechnology, School of Advanced Medical Sciences and Technologies, Shiraz University of Medical Sciences, Shiraz, Czechia; ^10^ Regional Centre of Advanced Technologies and Materials, Czech Advanced Technology and Research Institute, Palacký University in Olomouc, Olomouc, Czechia; ^11^ Department of Hematology, Faculty of Medicine, Tabriz University of Medical Sciences, Tabriz, Iran; ^12^ Toxicology and Chemotherapy Unit (G401), German Cancer Research Center, Heidelberg, Germany

**Keywords:** liposome, lipids, compounds, cholesterol, stability

## Abstract

Liposomes are essentially a subtype of nanoparticles comprising a hydrophobic tail and a hydrophilic head constituting a phospholipid membrane. The spherical or multilayered spherical structures of liposomes are highly rich in lipid contents with numerous criteria for their classification, including structural features, structural parameters, and size, synthesis methods, preparation, and drug loading. Despite various liposomal applications, such as drug, vaccine/gene delivery, biosensors fabrication, diagnosis, and food products applications, their use encounters many limitations due to physico-chemical instability as their stability is vigorously affected by the constituting ingredients wherein cholesterol performs a vital role in the stability of the liposomal membrane. It has well established that cholesterol exerts its impact by controlling fluidity, permeability, membrane strength, elasticity and stiffness, transition temperature (Tm), drug retention, phospholipid packing, and plasma stability. Although the undetermined optimum amount of cholesterol for preparing a stable and controlled release vehicle has been the downside, but researchers are still focused on cholesterol as a promising material for the stability of liposomes necessitating explanation for the stability promotion of liposomes. Herein, the prior art pertaining to the liposomal appliances, especially for drug delivery in cancer therapy, and their stability emphasizing the roles of cholesterol.

The article "Liposomes: Structure, Biomedical Applications, and Stability Parameters With Emphasis on Cholesterol" was retracted in 2023. Reasons: signs of a paper mill; concerns about the authorship.

## Introduction

Increasing advances in nanotechnology and nanoscience have raised great hopes in the field of biomedicine. Due to their unique, multifaceted and flexible properties, nanomaterials circumvents many challenges in diverse fields of medicine, including health, diagnosis, and treatment (Liu et al., 2020; Naskar and Kim, 2021), nanoliposomes being one of the most widely used nanoparticles in biomedicine. Liposomes are lipid bilayer spherical membranes that provide both hydrophilic and hydrophobic environments. Adjustability, flexibility, variety of ingredients, ease of functionalization, tunability of the number of layers/sizes, biocompatibility, and biodegradability have turned liposomes into incredible structures in medicine, especially drug delivery (Aguilar-Pérez et al., 2020; Trucillo et al., 2020; Kashapov et al., 2021), most notable use of these structures being in cosmetics and drug delivery. Consequently, various liposome-based products have been commercialized to date, with the approval from United States Food and Drug Administration (FDA) (Yuba, 2020; Barenholz, 2021). Liposomes, a type of lipid-based nanoparticle, have a great assortment each of which in turn offers unique properties. However, there are still barriers and challenges related to lipid nanoparticles, the most critical being their stability (Yu et al., 2021). In the present review, an attempt has been made to comprehensively deliberate liposomes in terms of structure, function, and stability starting initially with an introduction to lipid structures.

### Lipid Nanoparticles

Lipid molecules are one of the crucial elements of life and lipid-based nanoparticles comprise a broad range according to their application, components, shape, and fabrication methods; they possess numerous advantages over polymeric-based nanoparticles. Besides topical usage, agent delivery is ascribed to as a significant application of lipid-based nanoparticles. Being a physiological analog to the cellular membrane, liposomes have superior biocompatibility compared to polymeric-based nanoparticles, leading to a more acceptable biomedical application choices (Müller et al., 2000).

The article "Liposomes: Structure, Biomedical Applications, and Stability Parameters With Emphasis on Cholesterol" was retracted in 2023. Reasons: signs of a paper mill; concerns about the authorship.

As highly adaptable nanoparticles, lipidic nanoparticles can be deployed for a wide varieties of delivery with a bit of condescension. Liposomes and niosomes, as the phospholipid and amphipathic lipids constituents, respectively, are the most known lipid-based formulation. According to previous studies, liposomes could be engineered purposefully with favorable parameters. However, kinetic stability is the primary limitation of vesicular lipid-based nanoparticles, including liposomes (Battaglia and Ugazio, 2019). The most applicable lipid-based nanoparticles are presented in Table 1.

**TABLE 1:** Lipid-based structures.

Types	Structural features	Structural compositions
Liposomes (Pan et al., 2002; Thompson et al., 2006; Yavlovich et al., 2009; Chen et al., 2012)	1- Similarity to the cell membrane	DSPC- HSPC- DPPC-DOPEPC- EPCSPC-DMPC-DOPCCholesterol
	2- One or more concentric lipid bilayers enclosing an equal number of aqueous portions	
Emulsions (Pan et al., 2002; Cardenia et al., 2011; Lu et al., 2012)	1- Composed of two different phases, i.e., diffuse and continuous	PC- EPC – DOPC- DMPC DPPC- POPC- DSPC
	2- A liquid in liquid colloid structure	
	Composed of two immiscible liquids (usually oil and water). Liquid-liquid emulsions are mainly divided into two categories: water in oil (W/O) and oil in water (O/W) in which the oil phase and the aqueous phase form the continuous phase, respectively	
Micelle (Ashok et al., 2004; Faustino et al., 2011; Deng et al., 2012; Saadat et al., 2014)	1- The formation structure is based on the accumulation of diffused surfactant molecules in a colloidal liquid	PC- DSPE- DOPE- EPCGlycolic acid-lecithin
	2- Conventional and reverse micelles can be fabricated	
	Conventional micelles: hydrophobic tails assembled in the center of the micelles	
	Reverse micelle: the hydrophobic end is oriented towards the solvent, and the hydrophilic heads are gathered next to the center of the micelle	
Cochleates (Pawar et al., 2015; Mannino and Lu, 2018; Asprea et al., 2019)	1- Multilayered structures	PS and PC
	2- Composed of extensive and continuous two fat sheet layers	
	3- Stable structures with the two- valence phospholipid sediments of natural materials	
	4- It can be made of negatively charged phospholipids and a divalent cation	
	5- It can be used for delivering the hydrophobic and hydrophilic drug molecules; positively and negatively charged	
SLN (solid lipid nanoparticles) (Shah et al., 2007; Fang et al., 2008; Mehnert and Mäder, 2012)	1- Nanostructures with the solid core of the particle, which are mainly made of lipids, for delivering nucleic acids, proteins, and drugs	Tween 80- soybean phospholipids- SPC- squalene- precirol- PF68- glyceryl palmito-stearate
Nanostructured lipid carriers (NLC) (Müller et al., 2002; Müller et al., 2007)	1- SLN modified structures	1- Tween 80-phospholipids- glyceryl palmito stearate- glycyrrhizin- propylene glycol monostearate- lecithin, poloxamer 800, polyglyceryl-3methyl -glucose di-stearate, SDS, SDC, oleic acid, alpha-tocopherol/vitamin E, corn oil- squalene
	2- NLC, or oil-loaded SLN, contains lipid droplets that are partially crystallized and have a less regular or amorphous solid crystal structure to overcome the limitations of SLN	

**Note:** DMPC, Dipalmitoyl phosphatidylcholine; DOPC, Dioleoyl-sn-glycero-3-phosphocholine; DOPE, Dioleoyl phosphatidylethanolamine; DOPEPC, Dioleoyl phosphatidylethanolamine phosphatidylcholine; DPPC, Dipalmitoyl phosphatidylcholine; DSPC, Distearoyl-sn-glycero-3-phosphocholin; DSPE, Distearoyl-sn-glycero-3-phosphorylethanolamine; EPC, Ethanolamine phosphatidylcholine; HSPC, Hydro Soy phosphatidylcholine; PC, phosphatidylcholine; POPC, Palmitoyl-oleoyl-sn-glycero-phosphocholine; PS, Phosphatidylserine; SDC, Sodium deoxycholate; SDS, Sodium dodecyl sulfate; SPC, Sphingosyl phosphorylcholine.

The article "Liposomes: Structure, Biomedical Applications, and Stability Parameters With Emphasis on Cholesterol" was retracted in 2023. Reasons: signs of a paper mill; concerns about the authorship.

### Liposome Structure

Liposome structure has been initially described by the British hematologist, Alec D Bangham in 1961. From the terminology point of view, liposome consists of “Lipos” and “Soma,” attributed to fat and body, respectively. The cell membrane’s bilayer lipid structure has been determined using electron microscope images, proving their unmistakable resemblance to plasmalemma (Dua et al., 2012; Hashemzadeh et al., 2020a). Liposomes were recruited as a drug carrier for the first time in the early 1990s. It has since been concluded that the low percentages inclusion of lipid-bonded polymers (called polymer-lipids) in liposomes’ structure could increase blood circulation *in vivo*. Structurally, liposomes are concentric bleeder vesicles in which a membranous lipid bilayer surrounds an aqueous volume. Typically, the bilayer lipid membrane comprise phospholipids containing a hydrophobic tail and a hydrophilic head (Rovira-Bru et al., 2002).

According to the phospholipid’s properties, the final structure represents an amphiphilic feature (Dua et al., 2012). Due to the unique structure, both natural and synthetic phospholipids-based liposomes are considered vesicles or drug-carrying systems. The spherical or multilayered spherical design of the fabricated liposomes is highly reliant on the amount and the kind of lipid components. According to a concentric form, the bilayer lipid formation arrangement constitutes an equal number of water chambers (Chetoni et al., 2004; Choi and Maibach, 2005; Pavelić et al., 2005).

The article "Liposomes: Structure, Biomedical Applications, and Stability Parameters With Emphasis on Cholesterol" was retracted in 2023. Reasons: signs of a paper mill; concerns about the authorship.

In view of the utmost similarity to the cell membrane, the liposomes have been described as an appropriate membrane model to reveal the fundamental nature of cell membranes with assorted appliances (Wong et al., 2001; Laouini et al., 2012). The self-assembly of diacyl-chain phospholipids in aqueous solutions can form spherical bilayer structures referred to as liposomes. Because of encapsulating an extensive aqueous environment, liposomal structures can load almost any type of hydrophilic molecules (Lebègue et al., 2015; Vakili-Ghartavol et al., 2020; Wu et al., 2021). Liposome’s internal hydrophilic part can protect loaded drugs from the host body’s destructive factors that ultimately minimize the unwanted side effects. Besides the internal aqueous environment, hydrophobic substances can also be embedded between the lipid membranes or adsorb on the liposome surface (Xu et al., 2007; Silverman et al., 2013; Chen et al., 2014; Eloy et al., 2014; Jain et al., 2014). The essential liposome-like structures are presented in Table 2.

**TABLE 2:** Liposome-like structures.

Liposomes -like structure	Description
Niosome	Niosomes are attributed to carriers consisting of nonionic surfactants through cholesterol hydration (Sankhyan and Pawar, 2012; Puras et al., 2014; Arora, 2016)
Phytosome	Phytosomes are made from plant compounds. Phytosomes are lipid nanocarriers produced by phospholipids’ binding to polyphenols in organic solvents (Kidd, 2009; Jain et al., 2010; Pawar and Bhangale, 2015; Abd El-Fattah et al., 2017)
Virosomes	Virosomes are spherical shape structures with a mono/bilayer phospholipid-based membrane. The embedded central cavity of these structures is used to loading the therapeutic molecules such as nucleic acids, proteins, and drugs (Felnerova et al., 2004; Daemen et al., 2005)
BODIPYsome	The aza-BODIPY lipid is the building block that is self-assembled into a BODIPYsome vesicle structure capable of stable N.I.R. J-aggregation (Cheng et al., 2019)
DQAsomes	DQAsomes are vesicular structures composed of amphiphiles, decolinium (Zupančič et al., 2014; Weissig, 2015; Bae et al., 2018)
Archaeosomes	Archaeosomes is a new family of liposomes. They have been made of one or more ether lipids that are unique to the Archaea constitute domain. These types of structures are found in Archaeobacteria. Achaean-type lipids consist of archaeol (diether) and/or caldarchaeol (tetraether) core structures (Réthoré et al., 2007; Benvegnu et al., 2009; Kaur et al., 2016)
Ethosomes	Ethosomes are phospholipid nanovesicles. These structures are composed of flexible bilayers phospholipid, with a relatively high ethanol concentration (20–45%), glycols, and water. Transdermal delivery is considered the main application of the Ethosomes (Dayan and Touitou, 2000; Ainbinder et al., 2010)

The article "Liposomes: Structure, Biomedical Applications, and Stability Parameters With Emphasis on Cholesterol" was retracted in 2023. Reasons: signs of a paper mill; concerns about the authorship.

### The Packing Parameter

As described, liposomes are lipid-based structures that constitute one or more bilayer phospholipids which can encapsulate aqueous media. Liposome formation begins by dispersing phospholipids in water, leading to interactions between phospholipids and water (Anwekar et al., 2011), PP being a critical criterion determining the formation of liposome.

PP is described as the ratio between the cross-section of the amphiphile hydrophobic part (hydrocarbon chains of phospholipids or the hydrocarbon rings of sterols) and the cross-section of the hydrophilic part (the amphiphile head group). Liposome-forming lipids are considered amphiphilic structures with a PP of 0.74–1.0. In this regard, HSPC (PP: 0.8) and DSPE–PEG (PP: 0.487) have been addressed as liposome and non-liposome forming lipids, respectively. For DSPE-PEG, the low PP implied the presence of an extensive polar head group due to the large (45 mer) polyethylene glycol (PEG) moiety that prevents liposome-structure formation. The head group in this molecule is highly flexible (Nagarajan, 2002; Garbuzenko et al., 2005; Barenholz, 2016; Maritim et al., 2021). The most common phospholipids and cholesterol deployed to prepare liposomes with respect to their transition temperature (Tm) and molecular weights are presented in Table 3.

**TABLE 3:** The common compounds deployed to prepare liposomes.

Phospholipids	Molecular Formula	Electrical Charge	Tc (°C)	Mol. Wt.
Dilauryl phosphotidyl choline (DLPC) (Jung et al., 2005)	C32H64NO8P	−1	−1	633
Dimyristoyl phosphotidyl choline (DMPC) (Akabori and Nagle, 2015)	C36H72NO8P	0	23	678
Dipalmitoyl phosphotidyl choline (DPPC) (Jimbo et al., 2016)	C40H80NO8P	0	41	734
Dioleolyl phosphotidy l choline (DOPC) (Chibowski and Szcześ, 2016)	C44H84NO8P	-	−20	786
Dilauryl phosphotidyl ethanolamine (DLPE) (Benz et al., 2004)	C29H58NO8P	-	30.5	579.75
Dipalmitoyl phosphotidyl choline (DPPC) (Gullapalli et al., 2008)	C40H80NO8P	−1	41	734.053
Distearoyl phosphotidyl choline (DSPC) (Hashemzadeh et al., 2020b)	C44H88NO8P	0	58	790
Dioleolyl phosphotidy l choline (DOPC) (Attwood et al., 2013)	C44H84NO8P	0	−16.5	786
Dimyristoyl phosphotidyl ethanolamine (DMPE) (Li et al., 2015)	C33H66NO8P	0	50	635.85
Distearoyl phosphotidyl ethanolamine (DSPE) (Seo et al., 2011)	C41H82NO8P	0	-	748
Dilauryl phosphotidyl glycerol (DLPG) (Jacoby et al., 2015)	C30H58O10 PN a	−1	4	633
Dicetyl phosphate (DCP) (Chupin et al., 2002)	C32H67O4P	−1	-	546.85
Dioleoyl phosphatidyl ethanolamine (DOPE) (Evjen et al., 2011)	C41H78NO8P	-	−16	744
1,2-dioleoyl-3 trimethylammoniumpropane (DOTAP) (Caracciolo et al., 2005)	C42H80ClNO4	-	-	698.5
Dioleoyl phosphatidylserine (DOPS) (Okamoto et al., 2008)	C42H78NO10P	-	−10	788
Hydrogenated soybean phosphatidylcholine (HSPC) (Kitayama et al., 2014)	C42H84NO8P	-	52	762.1
Cholesterol (Bennett et al., 2009)	C27H46O	0	-	386.65354

The article "Liposomes: Structure, Biomedical Applications, and Stability Parameters With Emphasis on Cholesterol" was retracted in 2023. Reasons: signs of a paper mill; concerns about the authorship.

## Types of Liposomes

Liposomes are highly versatile compounds and they can be fabricated with various combinations, their diversity and properties vary in structure, size, shape, and surface properties. One of the classification types of liposomes is founded on their size and amount of layers, for example, unilamellar and multilamellar liposomes. They can be subdivided into four main categories based on structural parameters: multilamellar liposomes/vesicles (MLV), oligolamellar vesicles (OLV), multilamellar liposomes/vesicles (MVV), and unilamellar vesicles (ULV). Furthermore, the ULV can be divided into giant unilamellar liposomes/vesicles (GUV) groups, large unilamellar liposomes/vesicles (LUV), medium unilamellar vesicles (MUL), and small unilamellar liposomes/vesicles (SUV), and based on size (Walde and Ichikawa, 2001; Gabriëls and Plaizier-Vercammen, 2003; Wagner et al., 2006; Drulis-Kawa and Dorotkiewicz-Jach, 2010; Baykal-Caglar et al., 2012; Garg and K. Goyal, 2014).

Despite the aforementioned classification of various liposomes, many liposome characteristics cannot be deduced, including synthesis techniques or their applications. Since the introduction of liposomes as lipid-carrying structures, many methods have been proposed for their fabrication. Each has some advantages and disadvantages that can be exploited depending on the practical function. The process of liposome making strongly affects the final properties, so special attention should be paid to the construction method. Liposomes are referred to as a very miscellaneous structure in terms of their charge and size, the ultimate size and electrical charge of the fabricated liposome being highly reliant on the manufacturing method and the types of phospholipid deployed. In this regard, liposomes synthesis methods can be categorized as dehydration and rehydration (DRV), reverse phase evaporation (REV), particularly for SUL, OLV, and MLV liposomes, vesicles prepared by extrusion technique (VET), and frozen and thawed (FAT) for MLV preparation (Zhang and Pawelchak, 2000; Scott and Jones, 2001; Xia and Xu, 2005; Zaru et al., 2007; Akbarzadeh et al., 2013; Pradhan et al., 2015). Assorted liposome types, according to the fabrication methods, are presented in Table 4.

**TABLE 4:** Liposome classification based on the synthesis method.

Techniques	Features	Advantages	Disadvantages
Extrusion technique (Al-Remawi et al., 2017; Wang et al., 2017)	1- Different pore size filters depending on the need	-	-
	2- Producing LUV or nanoliposomes is based on the pore-size of the filters		
Sonication (Nasrabadi et al., 2016; Veneti et al., 2016; Yu and Tang, 2016)	1- The most widely used technique for the preparation and production of liposomes and nanoliposomes	-	1- Low internal volume/encapsulation efficiency2- Low ability to remove large molecules and metal pollution from the probe tip
	2- One of the most straightforward techniques to size reduction and producing nano-liposomes		
	3- Probe sonication and bath sonication are the main techniques		
Microfluidization[(Alizadeh et al., 2015; Yu et al., 2015; Davidson et al., 2016; Devrim et al., 2016; Saliba et al., 2016; Tabatabaei Mirakabad et al., 2016)]	1- This method is used in the pharmaceutical industry to produce liposomes and pharmaceutical emulsions	1- Possibility of producing a large volume of liposomes2- Ability to adjust the average size of the liposomes3- High efficiency (up to 70%)	-
	2- A chamber of microfluidizer contains a divided pressure stream		
	3- Recruiting microfluidizer		
	4- without potentially toxic solvents		
Heating method (Mozafari, 2005; Mozafari et al., 2007; Panahi et al., 2017; Hadavi et al., 2020; Khosravi-Darani and Sheida Aarabi)	1- It can be used for nanoliposomal production	1- It does not have the disadvantage of other methods, such as: Not using toxic solvents like ethyl ether, containing methanol and chloroform2- Not using high pressures	-
	2- Decreases the production time and cost on an industrial scale which has received much attention		
	3- Produce hollow micro-liposomes (HM-liposomes) that can be used as vectors in drug and gene transfer		
Freeze-drying (lyophilization) (Chen et al., 2010a; Franzé et al., 2018)	1- Based on removing water from products in the frozen state	-	-
	2- This step takes place at very low pressures		
	3- This method can solve the long-term stability problem of the solvent		
	4- The uses of trehalose can help liposomes retain as much as 100% of their original contents, so trehalose (a carbohydrate) in this method can be used as a freeze protectant		
REV (Otake et al., 2001; Kafle et al., 2020)	1- A one-step method for producing liposomes that do not make any toxic organic solvent	-	-
	2- This method can lead to the production of L.U.V.s with the diameters of 0.1–1.2 μm		
	3- Have a high ability to trap both water-soluble and oil-soluble substances		
Solvent dispersion method (Mozafari, 2005; Dua et al., 2012; Akbarzadeh et al., 2013)	Includes ether injection and 1- ethanol injection methodsAt the ether injection method, a solution of lipids dissolved in diethyl ether or ether/methanol mixture was injected gently into the aqueous solution. The temperature should be set at approximately 55–65°C, or the experiment should perform under reduced pressure. In later stages, under vacuum condition, ether is removed from the environment, and eventually, liposome will be fabricated		Ether injection method1- Heterogeneous nature of the synthesized liposomes (70–190 nm)2- Exposure of compounds to relatively high temperatures3- Exposure of encapsulated compounds to organic solventsEthanol injection method1- Heterogeneous products (30–110 nm)2- The fabricated liposomes are very dilute3- It is difficult to remove all ethanol from the environment due to the formation of azeotrope with water. Failure to completely remove ethanol from the reaction medium and formation of an azeotrope with water may lead to inactivation of biologically different activities
	2- ethanol injection method: In this method, ethanol’s lipid solution is rapidly injected into a vast excess of the buffer. At this point, The M.L.V.s are formed immediately		

Regarding the production of liposome, in addition to the fabrication method, drug loading should also be considered. In general, drug loading is performed *via* two standard procedures, passive and active loading, which affects the amount and quality of the loaded drug and some extent on the liposome properties. In the active loading method, known as the remote loading method, the drug molecules are loaded into the fabricated liposome. The pH gradient and electrical potential difference across the liposomal membrane are the most known underlying mechanisms dictating the active drug loading (Figure 1). The active loading method has provided various advantages over passive loading methods, including high efficiency and loading capacity, decreasing the loaded drug’s leakage, and reducing the drug’s shrinking during storage. Another outstanding feature of this method is the possibility of drug loading after carrier formation due to the use of the flexibility of constitutive lipid. It is also possible to prevent the degradation of the biologically active compounds during the preparative process (Barratt, 2003; Anwekar et al., 2011; Agrawal et al., 2012; Burton et al., 2015).

The article "Liposomes: Structure, Biomedical Applications, and Stability Parameters With Emphasis on Cholesterol" was retracted in 2023. Reasons: signs of a paper mill; concerns about the authorship.

**FIGURE 1:** The active and passive drug loading on the liposomes.

It has been well known that liposome characteristics are highly dependent on lipid composition. Surface charge, particle size, and the preparation method are among the most outstanding influenced features by lipid combination. Besides, the effective properties of bilayer structure, including rigidity, fluidity, and electrical charge, can be determined through bilayer component selection. In this regard, natural-based liposomes fabricated from unsaturated phosphatidylcholine species, including egg or soybean phosphatidylcholine, have provided bilayer structures with highly permeable and low stable properties. However, saturated-phospholipids-based liposomes such as dipalmitoyl phosphatidylcholine lead to rigid and almost impermeable bilayer structures (AllenLiposomes, 1997; Sahoo and Labhasetwar, 2003). The most common liposomal system, in terms of its composition constituent, are presented in Table 5.

**TABLE 5:** liposome classification according to composition constituents.

Types	Feature
Conventional liposome	Spontaneously self-assembled phospholipids (Neutral/negative charge) in an aqueous medium. The fabricated liposomes have surrounded an aqueous medium (Zhao et al., 2005; Zaru et al., 2007; Meure et al., 2008)
Fusogenic liposome (FL)	The liposomal system is based on reconstitute Sendai virus (Nakanishi et al., 2000; Kunisawa et al., 2005)
Cationic liposome	Liposomes containing the cationic lipid (Dokka et al., 2000; Radwan Almofti et al., 2003; Sioud and Sørensen, 2003)
Long circulatory liposome	The obtained products can improve tissues localization. These types of liposomes are liposomes with neutral high transition temperature (Moghimi et al., 2001; Awasthi et al., 2003; Metselaar et al., 2003; Moghimi and Szebeni, 2003)
P.H. sensitive liposome	These liposomes usually contain phosphatidylethanolamine (P.E.) and titratable stabilizing amphiphiles that become unstable under acidic conditions (Simões et al., 2004)
Immunoliposome	Long-circulating liposomes that may contain monoclonal antibodies or their fragments (Fab ') (Park et al., 2004; Hua, 2013)

## Application of Liposomes

As highly versatile nanoparticles, liposomes have been considered for many biomedical applications (Figure 2). Liposome as cholesterol and natural-non-toxic phospholipids-based spherical shape vesicles has provided many biomedical opportunities, especially for drug delivery ascribed to their biocompatibility, appropriate size, and suitable hydrophobic and hydrophilic character. Besides, the cosmetics industry has been vigorously affected by liposome formulations as they proposed many unique properties for drug carriers (Figueroa-Robles et al., 2020; Matole et al., 2020). On the other hand, the great potential application of liposomes should not be underestimated in the food and farming industries. Numerous studies have been conducting regarding liposome encapsulation to develop appropriate delivery systems to entrap unstable compounds. The ensnared invertebrate ingredients such as antimicrobials, antioxidants, hydrophobic, and hydrophilic compounds in liposome particles could be used to targeted delivery and prevent composition and functionality disruption (Benech et al., 2002; Shehata et al., 2008; Atrooz, 2011).

The article "Liposomes: Structure, Biomedical Applications, and Stability Parameters With Emphasis on Cholesterol" was retracted in 2023. Reasons: signs of a paper mill; concerns about the authorship.

**FIGURE 2:** Diverse biomedical applications of liposome-based structure.

The nanoliposome is a favorable particle to develop cancer drug delivery systems due to its unique properties, including biocompatibility, biodegradability, and hydrophilic and lipophilic drug loading capability. Liposome-based structures have owned the most commercial delivery systems worldwide. There is various ongoing research regarding improvement drug toxicity and specific targeting with liposomes (Akbarzadeh et al., 2013).

In view of the admirable properties mentioned for liposomes, it has been extensively studied in drug delivery to cancerous and tumor tissues *via* two main approaches in terms of design to target tumor tissues: passive targeting and active targeting (Figure 3). Passive targeting is reliant on the physiological characteristics of the tumor and the size of the nanoparticles. Cancer cells overexpress vascular endothelial growth factor (VEGF) due to their very high metabolism, which leads to excessive angiogenesis in tumor tissue. The vascular pores in the tumor tissue are larger than normal tissue, and the appropriate size of the liposomes enable them to circulate for a longer time in the circulatory system, so the anti-cancer drug nanosystem could target the tumor tissue (Zhu et al., 2017; Jeon et al., 2020; Liu et al., 2021). In addition, after the drug delivery system enters the cancerous tissue due to defects in the lymphatic system, the retention time of nanoparticles increases, which is not possible for the small drug molecules (Attia et al., 2019). In this method, the nanosystem is also coated with a biocompatible PEG polymer, which causes the escape of the reticuloendothelial (RES) system and increases the circulation time in the circulatory system; effect of PEG is through shielding liposomes from opsonization (Suk et al., 2016; Nunes et al., 2019).

**FIGURE 3:** Passive targeting and active targeting. Liposomes can be surface functionalized to dedicate stealth through PEGylation and to meliorate receptor-mediated endocytosis by utilizing targeting ligands such as antibodies, peptides, proteins, carbohydrates, Aptamer, and various other small molecules. PEGylation prolongs liposomal circulation half-life *in vivo*. Types of drugs based on whether they are hydrophobic or hydrophilic can be encapsulated into the aqueous lumen, incorporated into the lipid bilayer, or conjugated to the liposome surface.

The article "Liposomes: Structure, Biomedical Applications, and Stability Parameters With Emphasis on Cholesterol" was retracted in 2023. Reasons: signs of a paper mill; concerns about the authorship.

Despite the relatively good performance of passive targeting in increasing drug delivery to cancerous tissues, the optimum amount may still not reach the target tissue, or the drug may leak into normal tissues. Hence, researchers are using the active targeting method to enhance drug delivery to the target tissue. The basis of this method can be attributed to the functionalization of the liposome surface. Cancer cells need more nutrients because of their distinct metabolism. Therefore, some surface receptors are overexpressed on the surface of these cells. Targeted drug delivery to the cancerous tissue can be performed using this feature through specifically functionalizing liposome surface (Dana et al., 2020; Montaseri et al., 2020; Raj et al., 2021).

A comprehensive overview of liposomes’ applications in biomedicine is summarized in Table 6 according to the type of liposomes used.

**TABLE 6:** The use of liposome in biomedical applications.

Liposome type	Applications	Studies
Conventional liposome	Drug delivery	Improving the therapeutic index of encapsulated doxorubicin (Hilmer et al., 2004; Papagiannaros et al., 2006)
		Improving the therapeutic index of encapsulated amphotericin (Bern et al., 2006; Ellis et al., 2009)
		Liposomes have been used for sustained release cytarabine (Domínguez et al., 2005; Benesch and Urban, 2008)
	Cosmetics	Liposome has been recruited for‐ 4 ‐ n ‐ butyl resorcinol 0.1% cream encapsulation for the treatment of melasma (Huh et al., 2010)
		Liposomes have been used for skin wound healing application as antifibrogenic effects through IFN-alpha 2b encapsulation as cream formulation (Fuchsluger et al., 2006)
		Using liposomal hydrogel with polyvinylpyrrolidone iodine in the topical treatment of partial-thickness burn wounds (Homann et al., 2007)
	Vaccine adjuvant	NE and HBsAg in protein and DNA + protein have been entrapped into liposomes to induce immune response for hepatitis E and hepatitis B (Shrivastava et al., 2009)
		Lipid A-containing liposomes: A non-toxic adjuvant for the malaria sporozoite vaccine in humans (Alving et al., 2012)
		CAF01 liposomes as a mucosal vaccine adjuvant (Christensen et al., 2010)
	Sensors and Biosensors	Polydiacetylene liposome arrays for selective potassium detection (Lee et al., 2008)
		Immobilized-liposome sensor system for detection of proteins under stress conditions (Jung et al., 2007)
		Liposome to detect acute leukemia based on electrochemical cell sensor (Ghazizadeh and Neshastehriz, 2020)
	Vaccine therapy	BLP25 liposome vaccine to treat non-small cell lung and prostate cancers (North and Butts, 2005)
		P5 HER2/neu-derived peptide conjugated to liposomes containing M.P.L. adjuvant as an effective prophylactic vaccine formulation for breast cancer (Farzad et al., 2019)
		Liposomes containing interferon-gamma as an adjuvant in tumor cell vaccines (Van Slooten et al., 2000)
Fusogenic liposome (FL)	Labeling	Novel fusogenic liposomes for fluorescent cell labeling and membrane modification (Csiszár et al., 2010)
		Fusogenic liposomes for cell membrane labeling and visualization (Kleusch et al., 2012)
		Intracellular delivery of carboxyl coated CdTe quantum dots mediated by fusogenic liposomes (Lira et al., 2013)
	Gene transfer	Gene transfer with fusogenic liposomes containing vesicular stomatitis Virus G Glycoprotein (Shoji et al., 2004)
		Subcellular trafficking of antisense oligonucleotides and down‐regulation of BCL‐2 gene expression in human melanoma cells using a fusogenic liposome delivery system (Hu et al., 2002)
		Transferring maternally administered fusogenic liposome‐DNA complexes into monkey fetuses in a pregnancy model (Hirano et al., 2002)
	Drug delivery	Fusogenic liposomes to deliver mucosal insulin (Goto et al., 2006)
		Fusogenic liposomes containing diphtheria toxin fragment A to suppress tumor growth (Fang et al., 2005)
		Transferring antibodies and doxorubicin to the cytoplasm based on fusogenic liposomes for the metastatic treatment of breast cancer (Deng et al., 2017)
	Vaccine	Fusogenic liposome (F.L.) containing non-methylated CpG motif to increase antigen-specific immunity in mice (Yoshikawa et al., 2006a)
		Fusogenic liposomes (F.L.) can efficiently deliver exogenous antigen through the cytoplasm into the MHC class I processing pathway (Nakanishi et al., 2000)
		Fusogenic liposomes have the potential to be used as an effective vaccine carrier for peptide vaccination to induce cytotoxic T lymphocyte (CTL) response (Sugita et al., 2005)
	Vaccine therapy	Membrane fusogenic liposomes vaccine against melanoma that can produce both systemic immune and CTL responses (Qiang et al., 2004)
		Versatile cancer immunotherapy using vaccine of fusogenic liposomes containing tumor cell-lysate against murine B16BL6 melanoma (Yoshikawa et al., 2006b)
Cationic liposome	Gene delivery	Cationic liposomes to transmit human cystic fibrosis transmembrane conductance regulator (CFTR) gene to mouse models of cystic fibrosis (CF) (Lee et al., 2012)
		Cationic liposomes for co-delivery of small interfering R.N.A. and a M.E.K. inhibitor for enhanced anticancer efficacy (Kang et al., 2011)
		Trilysinoyl polyamide-based cationic liposomes for systemic co-delivery of siRNA and an anticancer drug [ (Shim et al., 2011)
	Drug delivery	Cationic liposomal doxorubicin (LPs-DOX) and paclitaxel (LPs-PTX) via electrostatic force to tumor cells (TRAMP-C1, B16) and HUVEC cells *in vitro* (Chen et al., 2010b)
		targeted delivery of cationic liposome-encapsulated paclitaxel (EndoTAG-1) for treating CNV (Gross et al., 2013)
		Cationic liposomes containing doxilagainst human SKOV-3 ovarian adenocarcinoma xenograft rat model (Jung et al., 2009)
	Vaccine adjuvant	Cationic liposomes containing mycobacterial lipids as Th1 Adjuvant (Rosenkrands et al., 2005)
		Cationic liposomes based on dimethyldioctadecylammonium and synthetic cord factor from *M. tuberculosis* (trehalose 6,6′dibehenate)—A adjuvant inducing both strong CMI and antibody responses (Davidsen et al., 2005)
		Cationic liposomes as a potent adjuvant for DNA vaccine of human immunodeficiency virus type 1 (Qiao et al., 2016)
	Vaccine therapy	Cationic liposomes as an antitumor autologous lewis lung cancer cell vaccine engineered to secrete mouse Interleukin 27 (Zhang et al., 2013)
		Cationic liposome-based synthetic long-peptide vaccines lead to strongly activate functional, antigen-specific CD8 + CD4 + T cells and induce *in vivo* cytotoxicity against melanoma and HPV-induced tumors in mice (Varypataki et al., 2017)
		Dendritic cells pulsed with tumor extract–cationic liposome complex increase the induction of cytotoxic T lymphocytes in mouse malignant glioma (Aoki et al., 2001)
Long circulatory liposome	Photodynamic therapy (PDT)	Glucuronatemodified (also known as long-circulating liposomes) liposomalized BPD-MA into Balb/c mice bearing Meth A sarcoma by PDT (Ichikawa et al., 2005)
		Anti-angiogenic PDT using long-circulating liposomes modified with peptide-specific to angiogenic vessels as a carrier for delivering photosensitizer to angiogenic endothelial cells (Ichikawa et al., 2004)
	Cancer therapy	Liposomes containing lipid derivatives of polyethylene glycol (sterically stabilized liposomes), known as long-circulating liposomes, were used to transfer doxorubicin to squamous cell lung carcinoma through specific antibodies attached to the liposome surface (Bakker-Woudenberg, 2002)
		Marqibo^®^:long circulating liposomes containing vincristine sulfate (Zhang et al., 2016)
		Long circulatory liposomes containing adriamycin were used in Colon 26 NL-17 carcinoma bearing mice and especially angiogenic site (Maeda et al., 2004)
	Gene delivery	pH-sensitive liposomes to transfer plasmid D.N.A. into mammalian cell lines (Chen et al., 2013)
		Encapsulation of a plasmid containing the *E. coli* chloramphenicol acetyltransferase gene in a pH-sensitive liposome and improvement of its transfection conditions (Torchilin, 2006)
		DNA entrapped pH-sensitive liposomes as a system for the transformation of tobacco mesophyll protoplasts (Hahn and Friedt, 2012)
pH-sensitive liposome	Gene delivery	PH-sensitive liposomes have been used as an intelligent system for the delivery of antisense oligonucleotides (Fattal et al., 2004)
		Anionic pH-sensitive liposomes were used as a delivery system for the smart delivery of antisense oligonucleotides (Fattal et al., 2004)
		pH-sensitive liposomes containing antisense oligodeoxynucleotide, ribozyme, and acyclic nucleoside phosphonate analogs for enhanced inhibition of HIV1 replication in macrophages (Düzgünes et al., 2001)
	Antibiotic Delivery	pH-sensitive liposomes to encapsulate gentamicin as an intracellular delivery system and improving its activity against intracellular pathogens (Cordeiro et al., 2000)
		pH-sensitive nystatin liposomes increased the antifungal activity against cryptococcus neoformans (Nasti et al., 2006)
		Endolysin LysRODI anti-staphylococcal encapsulation in pH-sensitive liposomes provides targeted delivery under mildly acidic conditions (Portilla et al., 2020)
	Proteins and peptides delivery	The pH-sensitive stealth liposome was used to deliver a therapeutic peptide to its nuclear site of action (Ducat et al., 2011)
		A pH-sensitive polymer-liposome-based antigen system was used as an interferon-γ gene delivery system lipoplex for efficient cancer immunotherapy (Yuba et al., 2015)
Immunoliposome	Drug delivery	Immunoliposomes can deliver high amounts of the 10B atoms into tumor cells and exert a cytotoxic effect by thermal neutrons (B.T.S. Thirumamagal et al., 2006)
		The dual peptides-modified liposomes loading VEGF siRNA and D.T.X. can inhibit glioma cell growth in a synergistic manner (Yang et al., 2014)
		Liposomes containing doxorubicin and NGR peptide targeting aminopeptidase N, a marker of angiogenic endothelial cells, were used to treat neuroblastoma (NB) in SCID mice (Pastorino et al., 2003)
	Diagnosis	Liposomes coated with polyethylene glycol and modified with monoclonal antibody 2C5 were used as contrast agents for the diagnosis and molecular imaging of tumor by SPECT/CT (Silindir et al., 2013)
		Reporter DNA encapsulated liposomes and surface modified with biotin-labeled polyethylene glycol (PEG) phospholipid can be used as a surrogate to quantify the target protein using real-time PCR (He et al., 2012)
		A liposomal immunosensor was used to monitor insulin and manage diabetes (Ho et al., 2006)
		An immunoliposome complex containing an anti-transferrin receptor single-chain antibody fragment (TfRscFv) decorating the surface and containing the contrast agent gadopentetate dimeglumine (“gad-d") was used to increase the sensitivity of detection of lung metastases (Freedman et al., 2009)
		IL-13-liposome-Gd-DTPA can cross the BBB and detect glioma at an early stage (Liu et al., 2016)

The article "Liposomes: Structure, Biomedical Applications, and Stability Parameters With Emphasis on Cholesterol" was retracted in 2023. Reasons: signs of a paper mill; concerns about the authorship.

### Advantages and Disadvantages of Liposomes

Like any other carrier, liposomes have provided some advantages and disadvantages, too. The benefits of liposomes have been mentioned briefly in this text. As amphiphilic and non-ionic structures particle, liposomes offer an exceptional opportunity to deliver both water and lipid-soluble drugs. This feature has a significant priority in the pharmaceutical industry to develop new formulations (Abdelkader et al., 2014; Joshi et al., 2016). On the other hand, their inimitable structure frame enables researchers to fabricate both sustained and targeted drug delivery systems through controlling permeability, rigidity, size, and surface functionalization (Daraee et al., 2016; Jain and Jain, 2016). Although liposomes can be administered through different routes, they are composed of biocompatible ingredients (Mansoori et al., 2012). One of the main limitations of drug distribution systems is the importance of biodegradable drug transport, which can be overcome through liposomal delivery that prevents drug oxidation (Manconi et al., 2016). It has been reported that liposomes can promote drug pharmacokinetics by eliminating and circulation life (Bhatt et al., 2018).

Despite all advantages, liposome-based structures have some limitation that prevents their widespread clinical use. The most significant obstacle is attributed to their physical and chemical stabilities (Bakker-Woudenberg, 2002). Among other essential impediments, low solubility in aqueous solutions (Li et al., 2019), short half-life time in body environment (Kshirsagar et al., 2005), high production cost (Noble et al., 2014), challenges in various tissue targeting due to the relatively large size of liposomes may cause (Santos et al., 2005), leakage and fusion of the loaded drugs (Joly et al., 2011), phospholipids oxidation and hydrolysis (Jain and Jain, 2016), rapidly detection by RES system (Daraee et al., 2016), and allergic reactions to some liposomal compounds (Mansoori et al., 2012), can be mentioned.

## Liposome Stability

One of the most critical challenges in liposome application is attributed to the relative instability in aqueous dispersions. The physical and chemical instability of liposomes can lead to unwanted side effects and efficacy reduction (Scrimgeour et al., 2005; Toh and Chiu, 2013); oxidation and hydrolysis are two primary mechanisms in the degradation of liposomes that cause chemical instability (Carlson et al., 2006; Jung et al., 2006; Frenzel and Steffen-Heins, 2015). The oxidation process is very probable due to free radicals in fatty acids as an intrinsic compound where unsaturated fatty acids are more susceptible than the saturated fatty acids to this mechanism (Anderson and Omri, 2004; Tan et al., 2016). In the presence of acid- or baseـ catalyst, this process can occur either at the 1-acyl or at the 2-acyl position, which subsequently leads to lysophospholipids through free fatty acids generation, eventually undergoing hydrolysis to free fatty acids and creating phosphoglycerols (Patel and Panda, 2012; Frenzel and Steffen-Heins, 2015). The combination of membrane bilayers, aggregation, reduced retaining of encapsulated materials, and alteration can be mentioned as the causes for physical instability in liposomes (Karmali and Chaudhuri, 2007; Shim et al., 2013; Rahdar et al., 2019).

The article "Liposomes: Structure, Biomedical Applications, and Stability Parameters With Emphasis on Cholesterol" was retracted in 2023. Reasons: signs of a paper mill; concerns about the authorship.

The administrated liposome fate and stability can be strongly affected by liposomes’ physicochemical characteristics, including bilayer membrane composition, size, rigidity, and charge (Portet and Dimova, 2010; Ghanbarzadeh et al., 2013; Ib and Corredig, 2013). The surface charge of liposomes can be positive, negative, or without electrical charge based on functional groups on liposomes’ surface at the environmental pH. As such, net-charge liposomes have represented the highest tendency to accumulate in the target tissue following systematic administration due to the reticuloendothelial system’s low clearance. On the other hand, cationic liposomes are often used to transport negatively charged nucleic acids (Xia and Xu, 2005; El-Samaligy et al., 2006a; Demetzos, 2008; Fujisawa et al., 2012). The methods used to prepare liposomes significantly affect physical properties, such as the coating of active compounds’ size and efficiency. Various phenomena such as aggregation and mixing can affect material properties, such as particle size and particle size distribution, attributed to the accumulation of liposomal particles. It has been reported that particle size reduction can be used for achieving bioactive compounds with optimal bioavailability due to increasing specific surface area (Campbell et al., 2001; Miao et al., 2002; Ulrich, 2002; Silva et al., 2011). The smaller the liposomal size, easier it is to cross the membrane, but it can affect the liposomal properties, including decreasing the amount and efficiency of drug loading and reducing liposome stability by increasing the surface energy. The smaller the particle size distribution, the more uniform is the liposomes’ size and the more similar would be the products’ overall characteristics (Marsh, 2001; Yamauchi et al., 2007; Drin et al., 2008).

Another critical factor affecting the stability of liposomes is referred to lipid composition. Studies have shown that controlling solute retention by liposomes and circulation half-life can be strongly affected by liposomal membrane fluidity and composition manipulation. One of the most critical barriers to prevent the transfer of liposomal drugs from the bench scale to the pharmaceutical market is their physical and chemical instability during production and storing. The mechanically robust and well-filled bilayers diminish the oxidizing and hydrolyzing agents that eventually improve the structure stability through size distribution (Kunzelmann-Marche et al., 2002; Liu and Krieger, 2002; López-Revuelta et al., 2006; Giulimondi et al., 2019); composition of the bilayer membrane is one of the influential and essential factors in liposome stability. The lipid selection during liposome fabrication should be commensurate with the carrier’s composition (Jiménez-Escrig and Sánchez-Muniz, 2000; Scheffer et al., 2005; Zhao et al., 2015; Ricci et al., 2016).

The article "Liposomes: Structure, Biomedical Applications, and Stability Parameters With Emphasis on Cholesterol" was retracted in 2023. Reasons: signs of a paper mill; concerns about the authorship.

### The Effect of Cholesterol on Liposome Membrane Stability

Cholesterol is an organic sterol molecule with amphiphilic nature. Structurally, this molecule has a hydroxyl group that can form hydrogen bonds with phospholipids and bulky steroid ring with a flexible carbohydrate. Cholesterol is a 27-carbon molecule found in the eukaryotic cell membrane and its concentration in the cell membrane is about 30–50 mol% of the entire lipid compounds. Various vital roles have been attributed to cholesterol, including membrane permeability regulation, elasticity and stiffness, and membrane strength. Cholesterol is the most used sterol in the formulation of liposomes which can prevent liposome aggregation and improve the liposomal membrane’s stability (Jiménez-Escrig and Sánchez-Muniz, 2000; Scheffer et al., 2005; Sun et al., 2007; Ricci et al., 2016; Trucillo et al., 2017).

In view of the spherical 3-D structure, liposomes have shown more realistic fluidity and cell membrane mobility than lipid monolayers. Sterols, such as ergosterol, stigmasterol, lanosterol, β-sitosterol and cholesterol, have been added to liposomes to modulate membrane fluidity and improve the stability of the phospholipids bilayer and decrease permeation of the encapsulated active compounds. The sterol molecule is located inside the phospholipid’s bilayer. The sterol carbohydrate tail at C17 intermingles with the hydrophobic fatty acyl chains, while the sterol hydroxyl group attaches to the hydrophilic head group of phospholipids (Socaciu et al., 2000; Sodt et al., 2015; Zhao et al., 2015; Giulimondi et al., 2019). Cholesterol plays a vital role in the liposome’s composition. It is one of the most critical structural components in the mammalian cell plasma membrane. It has been proven that the fluidity and permeability of the artificial vesicle are strongly affected by cholesterol through hydrogen binding to fatty acids that eventually lead to increasing the cohesiveness and mechanical strength. Cholesterol is a critical regulator of lipid bilayer dynamics, and it is essential for the normal functioning of the cells. The reduction of passive permeability to small molecules results from cholesterol interaction with membrane phospholipids, increasing the membrane cohesion. According to experimental studies, cholesterol adding to liposome bilayers can prevent lipid exchange that can be counted as an additional stabilizing effect (Sun et al., 2007; Ricci et al., 2016; Trucillo et al., 2017).

The article "Liposomes: Structure, Biomedical Applications, and Stability Parameters With Emphasis on Cholesterol" was retracted in 2023. Reasons: signs of a paper mill; concerns about the authorship.

### The Relationship Between Cholesterol and Transition Temperature

Another significant factor in the arrangement of bilayers in the liposome is the degree of saturation in phospholipids and the chain length. The presence of sterols such as cholesterol, β-sitosterol, and related plant sterols can lead to the pre-transition temperature peak’s disappearance. The gel-to-liquid crystalline phase Tm has been reported to decrease by addition of the sterols. It can be stated that the orientation of cholesterol in the lipid bilayer has a determinative effect on the reduction of head group accumulation. In the low Tm, cholesterol leads to the crystallization of the hydrocarbon chains into the inflexible crystalline gel phase. While in the high Tm, the rigid cholesterol molecule can limit the movement of the hydrocarbon chains. It can be concluded that, by increasing the sterol concentration, decreases the enthalpy of the main phase transition (Silva et al., 2011; Wu et al., 2012; Ricci et al., 2016).

For example, in the case of the PC molecule, it has been stated that cholesterol at concentrations of more than 25% leads to an order-liquid phase, which is essential for the mobility of membrane compounds; inferred that cholesterol at high concentrations causes the decouples of positional and conformational degrees of freedom of phospholipid molecules. On the other hand, at low cholesterol concentrations below 10%, its effect on the bilayer phospholipid is very different; only a slight decrease in the Tm, the main phase transfer occurs. This means that cholesterol at low concentrations cannot disrupt the crystalline order, nor can it ultimately induce the acyl chains in the liquid phase. Cholesterol, therefore, functions as a surfactant molecule, which causes the formation of lipid domains thus increasing the dynamic membrane heterogeneity (Trandum et al., 2000; Pinilla et al., 2020).

### The Role of Cholesterol in Retention of Drugs and Modulation of Phospholipid Packing

The cholesterol content has a critical role in drug retention as it implies its effect by raising the phospholipid packing, leading to bilayer permeability reduction to non-electrolytic and dielectrolysis solvents (Dos Santos et al., 2002; Johnston et al., 2007). It is believed that the underlying mechanism in a biological milieu may be related to the phospholipid and high-density lipoproteins exchange of the low-cholesterol or no-cholesterol content liposomes while in cholesterol-encompassing liposomes, the phospholipid motility has been limited that prevents lipoproteins loss (Kunzelmann-Marche et al., 2002; Liu and Krieger, 2002; López-Revuelta et al., 2006).

The article "Liposomes: Structure, Biomedical Applications, and Stability Parameters With Emphasis on Cholesterol" was retracted in 2023. Reasons: signs of a paper mill; concerns about the authorship.

The phospholipid packing, the membrane fluidity, and the surface charge of liposomes can be modulated and adapted by the cholesterol content, affecting the particle size, encapsulation efficiency, and final morphology (Zhao et al., 2015; Ohvo-RekilÃ et al., 2002). Studies have shown that cholesterol as a nonionic molecule has revealed interesting effects on the zeta potential, especially increasing the highest zeta potential of cationic liposomes. The proposed mechanism is reliant on the membrane structure transition and the molecular filling state for the cholesterol-induced charge boosting of cationic liposomes. Cholesterol can induce the phase transition from the crystalline state to the liquid-ordered (LO) phase (Lv et al., 2006; Aramaki et al., 2016). Increasing the amount of cholesterol content in the membrane of liposomes can increase the mean size of liposomes. Due to the hydrophobic nature, cholesterol structure can easily interact with the phospholipid hydrophobic acyl chain through hydrogen bonds and hydrophobic interactions. The ring structure of cholesterol is comparatively inflexible, and its presence stabilizes the protracted straight-chain arrangement of saturated fatty acids *via* van der Waals interactions (Lee et al., 2005).

### The Role of Cholesterol-Containing Liposomes in Plasma Stability

Cholesterol has a very significant effect on the structural stability of liposomes in plasma (Figure 4). It can reduce the interaction of liposomes with several proteins, leading to less susceptibility to phospholipase, reduce the phospholipid’s loss of high-density lipoproteins, change the membrane enzyme activities, inhibit digestion by macrophages, and inhibit fusion with specific cell types. By changing some liposome features through composition, mostly cholesterol modification, blood clearance and tissue distribution of intravenously injected liposomes can be expected. The cholesterol modification of liposomes has an inhibitory effect on the reticuloendothelial uptake. This modification reduces their interaction with several proteins and probably with serum components, which may affect liposomes’ tissue uptake (D’Avanzo et al., 2011; Johnstone et al., 2001; Moghimi and Patel, 2002). The cholesterol-based liposomal products are presented in Table 7.

The article "Liposomes: Structure, Biomedical Applications, and Stability Parameters With Emphasis on Cholesterol" was retracted in 2023. Reasons: signs of a paper mill; concerns about the authorship.

**FIGURE 4:** The liposome preparation and the role of cholesterol in its stability.

**TABLE 7:** Cholesterol-based liposomal products.

Drug compounds	Composition	The purpose of using cholesterol
Vitamin E (Samuni et al., 2000)	EPC + PUFA + cholesterol	1- Increasing the storage time by reducing physical and chemical changes: a- Decreasing the lipid-bilayer hydration
		b- Reduction in oxidative levels
5(6)carboxyfluorescein 5(6) (CF) (Liang et al., 2007)	DPPC + cholesterol	1- Increasing physical stability and reducing liposome deformity
Epirubicin (Wang et al., 2010)	CHCS + phosphatidylcholine + cholesterol	1- Physical stability
		2- Drug release
Doxorubicin (Zhao et al., 2007)	mPEG-DSPE + HSPC + cholesterol	1- Inhibiting aggregation through the steric barrier
		2- Prolonged blood circulation *in vivo*
CF (Abu-Dahab et al., 2001)	DPPC + LC-Biotin-DPPE + cholesterol	1- Enhancing the stability
Paclitaxel (Yang et al., 2007)	SPC + EPC + PE + DSPC + DPPC + HPC + cholesterol	1- Improving physicochemical stability
Vinorelbine (Semple et al., 2005)	SM + cholesterol	1- Improving drug retention
		2- Prolongation of plasma
		3- Circulation time
		4- Improving therapeutic activity
Curcumin (Chen et al., 2009)	DMPC + DMPG + cholesterol	1- Improving the bioavailability and efficacy of drug-containing liposomes
Vincristine (Liang et al., 2008)	PC + OQCMC + cholesterol	1- Good physical form
		2- Thermal stability
		3- Excellent solubility in water
		4- High effectiveness in drug encapsulation
Tenofovir (Xu et al., 2011)	DMPC + DPPC + DSPC+ DPTAP + cholesterol	1- Reducing the membrane permeability
Amphotericin B (Matsuoka and Murata, 2002)	POPC + EPC + FCCP + cholesterol	1- Preventing the formation of ion channels in the crystalline phase of the membrane of the liquid
		1- Inhibiting AmB-induced membrane permeability
Minoxidil (Mx) (López-Pinto et al., 2005)	α-DPPC + cholesterol	1- Increasing the drug-entrapment percentage, due to the stabilizing effect of cholesterol into the lipid bilayers
		2- An increase in the mean particle size
		3- Eliminating the phase-transition temperature (Tc) peak of DPPC and thus the range of the gel state of vesicles increased
		4- Preventing the partial dilution of the bilayers
		5- Decreasing permeability and making more rigid
CLX (celecoxib) (Deniz et al., 2010)	DSPC + cholesterol	1- Reduction of phase transition temperature (Tm)
		2- Encapsulation efficiency, loading, and releasing CLX decreased with the increasing cholesterol content
		3- Increasing drug retention
Acetazolamide (Hathout et al., 2007)	PC + holesterol + SA + DP	1- Increasing drug loading by 2- Increasing cholesterol
		3- Increasing Physical stability
		4- Increasing retained drug
Silymarin (El-Samaligy et al., 2006b)	Lecithin Soya + SA + DP + cholesterol	2- Adding cholesterol beyond a specific limit produced a decrease in encapsulation efficiency
Dithranol (Agarwal et al., 2001)	phosphatidyl choline + DCP + cholesterol	3- 1- Increasing entrapment efficiency of dithranol
Ciprofloxacin (Hosny, 2010)	PC + cholesterol	1- Optimal encapsulation efficiency by increasing a certain amount of C.H. content
		2- Improving prolonged drug
		3- Agent helping to control drug release

**Note**: CF, carboxyfluorescein; CLX, celecoxib; EPC, Ethanolamine phosphatidylcholine; PUFA, Polyunsaturated fatty acids; DPPC, Dipalmitoyl phosphatidylcholine; PEG-DSPE, Distearoyl-sn-glycero-3-phosphoethanolamine-Poly(ethylene glycol glycol, HSPC: Hydrogenated soybean phosphatidylcholine; LC-Biotin-DPPE, N((biotinyl)amino)hexanoyl)dipalmitoyl-l-α-phosphatidylethanolamine; SPC, Sphingosyl phosphorylcholine; PE, phosphatidyl-ethanolamine; DSPC, Distearoyl L-3-phosphatidylcholine; HPC, hydrogenated soybean phosphatidylcholine; SM, sphingomyelin; DMPC, dimyristoylphosphatidylcholine; DMPG, dimyristoylphosphatidylglycerol; PC, phosphatidylcholine; OQCMC, octadecyl quaternized carboxymethyl chitosan; DPTAP, 1,2-dipalmitoyl-3-trimethylammonium-propane; POPC, 1-palmitoyl-2-oleoyl-sn-glycero-3-phosphocholine; EPC, Egg yolk phosphatidylcholine; FCCP, carbonyl cyanid-*p*-trifluoro-methoxyphenyl hydrazone; α-DPPC, α-dipalmitoylphosphatidylcholine; SA, stearylamine; DP, dicetyl phosphate; DCP, Dicetyl phosphate.

The article "Liposomes: Structure, Biomedical Applications, and Stability Parameters With Emphasis on Cholesterol" was retracted in 2023. Reasons: signs of a paper mill; concerns about the authorship.

### The Optimum Cholesterol Concentration for Liposome’s Stability

The importance of cholesterol in liposome stability has been described earlier and schematically shows in Figure 3. However, the optimum concentration of cholesterol to attain a suitable formulation has not yet been elucidated. To make stable and regulated drug discharge means, lipids and cholesterol ratio screening arrangements in different studies can help. For the preparation of liposomes, some phospholipids are blended with varying molar ratios of cholesterol. The results of numerous studies have shown that the maximum amount of cholesterol that can be integrated into reconstructed bilayers is assumed to be ∼50 mol%. The most frequently used proportion is the 2: 1 ratio (e.g., two parts of lipids and one part of cholesterol) or 1: 1 ratio; although the underlying reasons for using these ratios is still unknown (Marsh, 2001; Liang et al., 2007; Briuglia et al., 2015).

The essential mechanisms of the liposomal interaction with cells according to both, *in vitro* and *in vivo* studies have been summarized as:

1- Particular interfaces with cell-surface components such as electrostatic bonds and imprecise interactions, including feeble hydrophobic bonds
2- Endocytosis caused by cells of the reticuloendothelial system (RES), comprising neutrophils and macrophages
3- Combination with the plasma cell membrane by inclusion of the lipid bilayer of the liposome into the plasma membrane (Akbarzadeh et al., 2013)

Adjusting cholesterol levels can be a very influential factor in controlling the liposomal stability. This factor can be crucial in designing liposomes for practical use in biological systems *in vivo* and *in vitro* (Epstein et al., 2008). The most important commercial liposomes are depicted in Table 8.

**TABLE 8:** Commercial cholesterol-based liposomes.

Commercial name	Composition	Type of drug	Application
LADR (small-sized liposomal Adriamycin) (Chen et al., 2005)	Cholesterol + egg phosphatidylcholine	doxorubicin HCl	Anti-Cancer
AmBisome (Dynarowicz-Łątka et al., 2003)	HSPC + DSPG + cholesterol	Amphotericin B	Anti-fungal
Doxil®/Caelyx®a (Wibroe et al., 2016)	HSPC + cholesterol + DSPE-PEG2,000	Doxorubicin	Anti-Cancer
Myocet™ (Collier et al., 2017)	EPC + cholesterol	Citrate conjugated doxorubicin	Anti-Cancer
Marqibo® (Silverman and Deitcher, 2013)	Sphingomyelin + cholesterol	vincristine sulfate	Anti-Cancer
Abelcet® (Husain et al., 2010)	DMPC + DMPG	Amphotericin B	Anti-fungal
DaunoXome® (Lowis et al., 2006)	DSPC + cholesterol	Daunorubicin	Anti-Cancer
Depocyt® (Phuphanich et al., 2007; Crommelin et al., 2020)	Cholesterol + triolein + DOPC + DPPG	Cytarabine	Anti-Cancer
Lipo-dox (Huang et al., 2018; Weng et al., 2019)	DSPC + cholesterol + PEG 2000-DSPE	Doxorubicin	Anti-Cancer
Visudyne (Barnes et al., 2010; Jain et al., 2016; Rizvi et al., 2019)	EPG + DMPC	Verteporfin	PDT
DepoDur (Peravali et al., 2014)	Cholesterol + Triolein + DOPC + DPPG	Morphine sulfate	Pain control and management

DSPG, Distearoyl-sn-glycero-3-phosphoglycerol.

## Clinical Trials

Unlike most nanoparticles, which encounter serious challenges in entering the clinic for various reasons, including safety issues, liposomes are well accepted in the clinic, first liposome-based drug being approved was Doxil^®^[(Anselmo and Mitragotri, 2015; Bulbake et al., 2017; Singh et al., 2020)], a liposome-based Doxorubicin formulation that has been FDA approved in 1995 for the United States market to treat ovarian cancer and AIDS-related Kaposi’s sarcoma. Subsequently, various other liposomal-based drugs have been commercialized, such as DaunoXome^®^, for the delivery of daunorubicin, approved in 1996 to manage advanced HIV-associated Kaposi’s sarcoma and several different formulations (Khadke et al., 2020).

The article "Liposomes: Structure, Biomedical Applications, and Stability Parameters With Emphasis on Cholesterol" was retracted in 2023. Reasons: signs of a paper mill; concerns about the authorship.

Currently, many efforts are underway to develop lipid formulations for entry in to the clinics in various fields. To examine the clinical phase studies of liposome-based structures, the term “liposome” was searched from the PubMed database pertaining to various studies related to the clinical phases in the last year. In one study, the effect of liposomal amphotericin B formulation as an antifungal agent was investigated in patients with hematological malignancies with neutropenia and persistent fever (Yoshida et al., 2020). Because fungal infections subsequent to the chemotherapy in patients with neutropenia are considered a severe complication, and as the use of common antifungal drugs is highly toxic, so eliminating this life-threatening complication is very important. The usage of 3 mg/kg/day liposomal amphotericin B concentration for patients was compared with itraconazole; results showed no difference between the liposomal amphotericin B and itraconazole regarding the efficacy and safety in antifungal therapy in hematological malignancy patients (Yoshida et al., 2020).

Liposomal compounds are known to be very effective in treating cancer. Recently, another liposomal system has been proposed for the treatment of acute myeloid leukemia wherein the Vyxeos liposome in phase III clinical was examined. This liposomal system comprise two different topoisomerase II inhibitors known as daunorubicin and cytarabine, which included 1 and 0.44 mg in every 1 unit of liposome formulation. The study was performed on elderly patients with untreated acute myeloid leukemia where a higher survival rate for patients treated with the liposomal formulation was discerned than for standard chemotherapy, although some side effects have been reported for the use of this formulation (Tzogani et al., 2020).

## Conclusion

Health and medical issues and problems have always been one of the main areas of interest for scientists. Applying new methods for solving medical problems requires introducing new and efficient materials and tools that address related questions and issues. Liposomes have been extensively studied since their introduction, and their potential biomedical use has been well demonstrated. The unique properties of liposomes, including biocompatibility, biodegradability, amphiphilic nature, low toxicity, non-ionicity, sustained release, and active targeting, have made them one of the most widely used nanoparticles. Currently, the most commercialized nanoparticles in the field of drug delivery and cosmetics are related to liposomes. However, they still have some shortcomings that need to be addressed for clinical and pharmaceutical use. As mentioned earlier, since Doxil^®^ introduced in 1995, many efforts have been made to bring these versatile nanomaterials to the clinic; however, their structure still needs to be optimized to reduce some complications. One approach to increase liposomes’ efficiency, especially concerning cancers therapy, is the use of RGD which can be anchored to liposome surfaces or *via* self-assembly means (Cheng and Ji, 2019). This strategy has been proposed to reduce the side effects of liposomal drugs, as the clinical trial sometimes suffers from, including acute infusion reaction and hand-foot syndrome (HFS). Hence future studies must include new procedures to reduce safety problems (He and Tang, 2018; Cheng and Ji, 2019). Since varying combinations of liposomes can provide unique and distinctive properties, exciting suggestions have been propositioned in the field of novel drug delivery systems, such as nose-to-brain direct drug transport using liposome formulation based on DTE and DTP ingredients (Hong et al., 2019).

The article "Liposomes: Structure, Biomedical Applications, and Stability Parameters With Emphasis on Cholesterol" was retracted in 2023. Reasons: signs of a paper mill; concerns about the authorship.

However, one of the most critical challenges that liposomes encounter is their physical and chemical instability. Various factors such as environmental conditions, manufacturing method, components characteristics, lipid type, and the absence or presence of cholesterol affect liposomes’ stability. The vital need for the development of liposomes with high stability significantly impacts their clinical application. Cholesterol has been shown to increase liposome stability through various mechanisms, including increased retention time, modulating phospholipid packing, Tm, and plasma stability. However, the optimal amount of cholesterol has not yet been identified. Future field research should be based on the principle of finding the optimal amount of cholesterol in liposome production. Notably, cholesterol still tend to maintain membrane’s fluidity as its concentration is increased and decreased. Therefore, the amount of cholesterol and the type of liposome constituents need further investigation. In this context, simulation and computational studies may prove to be very helpful. Hashemzadeh et al. (2020a) have investigated DSPC and DPSM effect on liposome stability through a simulation study which revealed that DSPC preserves its structure shape due to the cylindrical geometric structure and small-size head group, while the DPSM was causing liposome turnover into micelle structure because of its conical geometric design with the larger head group. Such studies regarding cholesterol’s effect on liposome stability *via* simulation investigations would be highly desirable.
